RETRACTED

# Clinical Observation of MRI Scanning Combined with Clinical Nursing for Surgical Breast Cancer Patients

**DOI:** 10.1155/2022/6863281

**Published:** 2022-05-17

**Authors:** Huan Zhang, Yanan Yin, Wenjing Tao, Ling Liu

**Affiliations:** ^1^Breast Cancer Center, Chongqing University Cancer Hospital Department, Chongqing 400030, China; ^2^Department of Medicine, Chongqing University Cancer Hospital Department, Chongqing 400030, China

## Abstract

The aim of this study was to explore the application effect of perioperative nursing care for patients with breast cancer. In this paper, 100 breast cancer patients with lymphatic spread treated by breast surgery in September 2019 to December were selected as the evaluation objects. They were divided into two groups according to preoperative imaging examination, 50 cases in each group. Group A was examined by B-ultrasound before axillary lymphadenectomy, group B was examined by MRI before axillary lymphadenectomy, and group C was examined by B-ultrasound and MRI before axillary lymphadenectomy. The facts in the three groups of disease findings were compared. Compared with the control group, the proportion of negative emotions (such as stress and depression) in the control group decreased (P<0.05). The decrease in blood cortisol was higher than in the control group (*P* < 0.05). Improving the existing cancer surgery can improve the patient's heart rate and reduce blood cortisol so as to improve the patient's joint function and quality of life. The difficulty of nursing patients will also be reduced, which is medically necessary.

## 1. Introduction

Breast cancer is one of the most common cancers in the world. According to the statistics, in 2012, an estimated 1.7 million new cases of leukemia were registered worldwide, and more than 520,000 people died of leukemia. In China, more than 270,000 new cases are reported each year, making it the number one cancer for women and the sixth leading cause of death for women. Studies show that by 2050, 3.2 million people worldwide will be diagnosed with breast cancer each year [1]. The incidence rate and mortality rate of breast cancer in China are lower than the world average. However, with the improvement of people's living standards and the change of lifestyle, the growth rate of breast cancer is particularly significant and tends to be younger. Surgical treatment has always been the most effective and most important treatment for breast cancer. There are many types of operations, and radical mastectomy is the most important way of operation. As the excision of breast tissue is too large, it will seriously affect the quality of life of patients and bring inconvenience to patients. In recent years, neoadjuvant chemotherapy (NAC) has been used more and more in the treatment of breast cancer. In particular, for locally advanced breast cancer, NAC has become the standard treatment. NAC can not only reduce tumor volume by preoperative chemotherapy but also eradicate metastatic lymph nodes and reduce the grade of cancer, thereby increasing the breast preservation probability, reducing the axillary lymph node dissection rate, avoiding some patients undergoing radical mastectomy, and improving the survival rate and quality of life of patients [2]. There are many ways to evaluate the effectiveness of breast cancer after NAC. These include breast routine physical examination, breast ultrasound, mammography, breast magnetic resonance imaging (MRI), breast positron emission tomography (PET/CT), and postoperative pathological examination. Although there are many clinical studies aimed at determining the best examination method, there is still no unified view so far. Postoperative pathological examination has always been regarded as the “gold standard” of diagnosis. For the traditional anatomical imaging methods, such as breast ultrasound and breast molybdenum target, it is difficult to distinguish between fibrotic tissue and residual tumor tissue, so their clinical use is very limited. Some studies show that breast MRI has obvious advantages, as shown in Figure 1. Therefore, many clinical workers praise breast MRI. However, some studies believe that breast MRI may overestimate or underestimate the size of residual tumors [3, 4]. In recent years, breast PET/CT imaging has increasingly been used to evaluate tumor responses to NAC breast and post-NAC cancers. As a functional metabolic imaging method, PET/CT can detect leukemia changes immediately after NAC, thus allowing early diagnosis of NAC function. The purpose of this study was to investigate relevant data and compare the accuracy of MRI and PET/CT scans to measure the response of leukemia to NAC by metascreen.

RETRACTED

## 2. Literature Review

The relevant research results of Goda et al. showed that, compared with nonmetastatic lymph nodes, the enhancement peak time of metastatic lymph nodes was significantly prolonged, the peak enhancement degree and maximum rise rate were decreased, and the clearance rate was slightly increased [5]. Zhang et al. studied axillary lymph nodes by DCE-MRI with reference to the research method of breast mass. The results showed that the proliferation of malignant tumors is usually of III type and that the predisposition curve of the malignant tumors is usually of the hom or hom type. There was a significant difference between them (*P* < 0.05). In breast cancer, the time signal used to curve the axillary metastatic lymph node is similar to that of primary cancer [6]. Zhuang et al. studied the breast cancer patients who underwent MRI enhanced scan. According to the morphological changes of lymph node inhomogeneity and lymph node volume (diameter >1.5 cm or 50% of the contralateral lymph node diameter), the sensitivity and specificity of lymph node metastasis were 86.2% and 95.3% [7], respectively. Saha et al. think that breast cancer (mammarycancer) is the most common malignant tumor in women. The incidence rate of this disease is 7–10% of all kinds of malignant tumors in the body. It has become the main cause of physical and mental health of women. The etiology of breast cancer has not yet been fully elucidated. However, many studies show that breast cancer may be related to the long-term stimulation of exogenous or endogenous estrogen, viral, genetic and family history, breast atypical hyperplasia, nutritional factors, and radiation lines, besides breast cancer [8]. Li et al. believe that breast cancer most commonly occurs in women aged 40–60 years, and the incidence rate of menopausal women is higher. It is the most common malignant tumor that usually occurs in breast glandular epithelial tissue. Its clinical manifestations include nipple changes, breast lumps, breast skin and contour changes, lymphadenopathy, and so on. It seriously affects women's physical and mental health and even endangers their lives. With the development of modern science and technology, the auxiliary examination of the disease includes breast molybdenum target, breast B-ultrasound, and dynamic enhanced nuclear magnetic resonance [9]. Zhao et al. believe that MRI is the imaging method with the highest resolution of soft tissue, which has many advantages over B-ultrasound and X-ray, and it is more reliable in the diagnosis of multicentric lesions. The specificity and sensitivity were more than 90%. Tumor microvessel distribution data can provide more tumor treatment response and functional parameters. MRI was not affected by dense breast, deep side, and high position. The image can be cut in any plane, which can clearly show the small tumor. However, it is not applicable to patients with metal in their body [10]. Saeed et al. believe that the important factor determining the quality of diagnosis is a good MRI image. The image quality is not only related to the setting of machine and scanning parameters but also closely related to the patient's good attitude and cooperative attitude. Therefore, taking appropriate nursing measures before, during, and after the examination is of great significance to ensure the quality of magnetic resonance image and diagnostic effect [11]. Rosenberger et al. believe that the general nursing, psychological nursing, and signing examination consent before the MRI scan can enable patients to have a thorough understanding of the examination mode before scanning, eliminate the patients' nervousness, and accept the examination with a good attitude. The posture guidance during the examination can make the patient maintain a correct and comfortable examination posture and ensure the formation of good magnetic resonance images. The psychological nursing in the process can enable the medical staff to quickly understand the psychological changes of the patient and accurately grasp any changes during the examination, while the injection drug nursing can ensure the correct and rapid injection of drugs and ensure the image quality. Routine nursing and health guidance after examination can understand the possible adverse reactions of patients at the first time and provide valuable suggestions for patients' future lifestyle and habits, so that patients can find the condition in time and seek medical treatment immediately [12]. MRI scanning plays an extremely important role in the diagnosis and treatment of breast diseases, but this method takes a long time, has a special body position, and often needs dynamic enhancement. Therefore, the active cooperation of patients is particularly important, which improves the requirements of clinical nursing. This article summarizes the nursing experience of patients with breast cancer MRI scan.

RETRACTED

## 3. Data and Methods

### 3.1. General Information

In the study group, the proportion of postoperative stress, depression, and other negative thoughts was lower than that in the control group (P < 0.05). Before MRI scanning, all cases in this group had obtained the results of ultrasound or X-ray molybdenum target examination, and all cases were confirmed by pathology after MRI scanning [13].

### 3.2. Inspection Method

The control group received routine B-ultrasound examination of breast and bilateral axillary before operation, and the study group received B-ultrasound combined with MRI before operation. B-ultrasound examination: la523 is used, and the probe frequency is 4–13 mhz. The patient was in supine or lateral position, and then the examination site was fully exposed. The morphological characteristics and blood supply of the lesion were observed by routine two-dimensional and color Doppler ultrasonography. Criteria for B-ultrasound suspicion of lymph node metastasis are as follows: lymph nodes are round; abnormal hilar structure disappeared; abnormal thickening of cortex and >3 mm; the shortest diameter >5 mm; MRI scanning: the instrument adopts a 1.5 T special MRI scanner for breast, with a layer thickness of 1.1 mm, a matrix of 360 × 360 × 128, and an interval of 0 mm. The fat suppression technology is used for four rounds of dynamic enhancement scanning. The contrast agent GG DTPA, with a dose of 0.2 mmol/kg, was injected through the dorsal vein mass of the hand with a high-pressure syringe at a flow rate of 2.9 ml/s. Criteria for suspected lymph node metastasis under MRI are as follows: round shape; abnormal thickening of cortex or abnormal enhancement after enhanced scanning; the shortest diameter >5 mm; and abnormal or disappearance of lymphatic hilus structure [14].

RETRACTED

### 3.3. Nursing Methods

1. Preexamination nursing. ① General nursing: before the examination, the nursing staff should introduce the environment and equipment of the examination room and the importance of the examination for the diagnosis of the disease to the patients in detail, and inform the patients that the magnetic resonance equipment will have a large noise under the normal working state, so that the patients have a certain psychological preparation. Assist the patient to remove metal objects (such as dentures, necklaces, rings, earrings, bras, watches, and mobile phones) from the body before scanning, wear light clothes and empty the, urine. Strictly grasp the patient's past medical history, whether there are contraindications for entering the examination room such as epilepsy and mental disease, and describe in detail the purpose of using the contrast agent, pharmacological effect, metabolism, and possible adverse reactions to the patients who need enhanced scanning. ② Psychological nursing: because breast cancer patients are all women and their location is special, according to the psychological characteristics of breast cancer patients, nurses should treat patients with initiative, enthusiasm, and sincerity when they first contact with them, patiently answer questions raised by patients, and try to provide the help they need. For patients with excessive tension and anxiety, we should enlighten them with appropriate methods and attitudes to adjust their mental and physical state. For patients who do not understand their condition, they should be cautious and take protective medical measures to ensure the smooth progress of MRI scanning process. At the same time, we should explain to the patients that the medical staff always pay attention to the whole examination process, so as to eliminate their ideological burden. ③ Sign the examination consent form: the nursing staff should carefully explain the general process and precautions of the examination to the subject and his family members, and ask the patient whether he has a history of allergy before taking the medicine. If he has a history of allergy, he should be cautious or not use the medicine. Inform family members that the probability of adverse reactions is low. Then ask the examinee and his family members to sign the examination consent, which can eliminate the patient's tension to the greatest extent and actively cooperate with the examination. At the same time, prepare various rescue drugs and rescue facilities [15].
2. Nursing during examination. ① Posture guidance: the nursing staff should remove the body phase control front ring on the scanning table and place the special double ring polar array breast coil on the scanning table to guide the patient to maintain the prone position, open the clothes, the bilateral breast naturally hangs in the hole of the coil, and pad soft pillows on the patient's feet, knees, and head to maintain posture and support the body. Because the patient's upper body is exposed, a thin quilt can be used to cover the body. ② Psychological nursing: during the scanning process, the nursing staff should closely monitor and observe the patient's situation. During the scanning interval, they can appreciate and affirm the patient's early cooperation through the intercom system, encourage them to continue to adhere to a reasonable posture, do not move their body, and avoid coughing, so as to prevent motion artifacts. Inform them that it is very important to maintain postural coordination when injecting high-pressure contrast medium. When injecting drugs, the fear caused by local pressure, cold feeling, swelling, and pain should be enlightened and informed in time. This phenomenon is normal. Don't worry. For patients with excessive tension, their families can be arranged to provide close care so that patients can eliminate psychological problems and fully feel the care of their families. ③ Injection drug care: the nursing staff should check whether the disposable intravenous infusion needle and the extension tube of the high-pressure syringe are connected tightly, whether the exhaust of each connection port of the high-pressure syringe is tightened, and guide the patient to hold the connection, first try to inject about 5 ml of normal saline, observe whether there is pain and leakage at the injection site, and ask the patient whether there is a cold feeling in front of the scalp needle. Medical staff should be agile and skilled in injection operation to avoid repeated operation [16].
3. Postexamination nursing. ① Routine nursing: after the examination, the nursing staff should timely ask the patient if there is any discomfort, pull out the disposable intravenous infusion needle, and guide the patient to press the needle eye for 5 min without kneading. Asked the patient not to leave immediately and observe the adverse reactions after medication. If there are discomfort symptoms such as dizziness, nausea, vomiting, and palpitation, corresponding nursing measures shall be taken in time. After confirming that the patient is not unwell for more than 30 minutes, the patient can be notified to leave, and the patient should be informed to drink more water to accelerate the excretion of drugs from the kidney. ② Health guidance: give appropriate health guidance to patients, tell them to carry out breast self-examination regularly, often carry out physical exercise, take fast walking and jogging as appropriate, prolong sleep time, and maintain abundant energy. Choose nutritious and healthy food, eat more fresh fruits, vegetables and other coarse fiber food, prevent constipation, avoid drinking and smoking, control body mass, and drink less coffee. Keep the spirit happy and calm, and avoid long-term stress and mental tension. Those who have not given birth are encouraged to give birth before the age of 30, and the lactation period is preferably more than half a year.

RETRACTED

## 4. Experimental Results and Analysis

### 4.1. Results

Comparison of B-ultrasound and MRI scanning results with postoperative pathological results showed that the coincidence rate between preoperative examination and postoperative pathological confirmation results in the study group was 95.56%, and the diagnosis coincidence rate in the control group was 77.78%. The difference between the two groups was statistically significant (*P* < 0.05, refer to Figure 2).

#### 4.1.1. Comparison of Misdiagnosis and Missed Diagnosis between the Two Groups

There was no misdiagnosis in the study group, two cases were missed, and the missed diagnosis rate was 4%. In the control group, three cases were misdiagnosed, the misdiagnosis rate was 6%, and seven cases were missed, and the missed diagnosis rate was 14%. The difference between the two groups was statistically significant (*P* < 0.05, refer to Figure 3).

#### 4.1.2. Comparison of Changes in Prenatal Care between the Two Groups

In the study group, the proportion of postoperative stress, depression, and other negative thoughts was lower in the study group. control (*P* < 0.05). group. (*P* < 0.05). See Figures 4 and 5.

As shown in Figure 6, the treatment satisfaction and cooperation of the two groups were compared.

MRI images of sick patients and healthy people are shown in Figure 7.

Comparison plot of ultrasound findings of healthy and diseased patients is shown in Figure 8.

### 4.2. Discussion

Breast cancer is a common female malignant tumor. It accounts for 10% of all kinds of malignant tumors in the whole body, and the incidence rate of female diseases is only inferior to that of uterine cancer. Breast cancer is prevalent among women aged 40–60 years. The risk of breast cancer is higher in women with high risk factors. The major risk factors for breast cancer include menarche age, menopause age, first pregnancy age, postmenopausal estrogen supplement, oral contraceptives, diet, weight gain, and so on. Imaging techniques such as B ultrasound and MRI scanning play an important role in the clinical diagnosis and treatment of breast cancer [17, 18]. Radical mastectomy is a relatively ideal treatment for breast cancer patients. It can improve the patient's condition to a certain extent and has a good therapeutic effect. The results of preoperative axillary lymph node status evaluation are directly related to the choice of follow-up treatment and affect the evaluation of disease prognosis to a certain extent. Therefore, preoperative evaluation of axillary lymph node status is very important for breast cancer patients. Ultrasonography is the preferred imaging method for breast diseases. Because of its low cost, no trauma, and no radiation, it can accurately determine the physical properties of breast masses and further analyze benign and malignant lesions. It is an indispensable technique for diagnosing breast cancer and axillary lymph nodes. However, conventional ultrasound cannot distinguish the benign and malignant [19, 20] from axillary lymph nodes sometimes. According to this study, the overlap between preoperative diagnosis and postoperative diagnosis was 95.56% in the study group and 77.78% in the control group. The differences between the two groups were significant (*P* < 0.05). The research team did not make a wrong diagnosis. The two cases are incomplete and 4% were undetected. In the control group, three people were misdiagnosed, and the misdiagnosed rate was 6% Seven people with disabilities were missed, and the missed diagnosed rate was 14%. Significant differences (*P* < 0.05) between the two groups suggest that a combination of preoperative breast ultrasound and MRI can be used to measure the incidence of axillary lymph nodes in patients with leukemia, to achieve better results, and to improve outcomes in advance, which is always consistent with current research to identify, diagnose, and prevent misdiagnosis of postoperative disorders [21]. MRI scanning has no radiation damage, has good spatial resolution and soft tissue resolution, and has high sensitivity in the diagnosis of breast cancer. It can largely improve the early resolution of breast cancer and improve the diagnostic accuracy. Therefore, breast MRI scanning has been widely used in clinic with its unique advantages and has been widely concerned by clinicians and imaging doctors [22]. In short, in clinical practice, corresponding examination methods should be selected according to the actual situation of patients to maximize the diagnostic accuracy and provide valuable reference basis for clinical diagnosis and treatment [23–26].

RETRACTED

## 5. Conclusion

The breast cancer MRI scanning before, after, and after the patient care not only increased the patient's awareness of breast cancer but also enhanced communication between nurses and patients, to ensure the harmony between nurses and patients and reduce the patient's bad mood, so that patients' satisfaction with clinical nursing work significantly improved. In this group of breast cancer patients, through reasonable and effective nursing measures, the quality of MRI images can be improved, the incidence of adverse reactions can be reduced, and the anxiety of patients can be significantly reduced. In conclusion, effective breast cancer MRI scanning patients' nursing strategies can significantly improve the quality of MRI images, reduce the recurrence rate of negative emotions, and make breast cancer patients self-confidence in examinations and improve their quality of life.

## Figures and Tables

**Figure 1:** Flowchart of MRI scan for breast cancer patients.

**Figure 2:** Comparison of ultrasonography and MRI results with postoperative pathological results.

**Figure 3:** Comparison of misdiagnosis and missed diagnosis between the two groups.

**Figure 4:** Comparison of perioperative mood changes of patients in the study group (MeanSD).

**Figure 5:** Comparison of perioperative mood changes of patients in the control group (MeanSD).

**Figure 6:** Comparison of treatment satisfaction and cooperation between the two groups.

**Figure 7:** Plot of MRI images of sick patients compared with MRI images of healthy people.

**Figure 8:** Comparison of ultrasound findings of healthy and diseased patients.

## Data Availability

The data used to support the findings of this study are available from the corresponding author upon request.
